The article "The Ecological Consciousness of Natural Writing in British and American Romantic Literature" was retracted in 2023. Reasons: unreliable results or conclusions; concerns about the data; concerns about the peer review; concerns about the citations.

# The Ecological Consciousness of Natural Writing in British and American Romantic Literature

**DOI:** 10.1155/2022/8233269

**Published:** 2022-08-11

**Authors:** Yanrui Jin

**Affiliations:** Foreign Languages Department, Shanghai University of Finance and Economics Zhejiang College, Jinhua, Zhejiang 321013, China

## Abstract

The ecological crisis made the British and American ecological literature develop rapidly in the 20th century ecological thought. As a unique literary style that expresses the relationship between nature and man, British and American ecological literature has a far-reaching romantic tradition, and returning to nature is its eternal theme and dream. The study of the romantic tradition of British and American ecological literature has important implications for the development of ecological literature and ecological criticism. British and American romantic writers wrote their own ecological consciousness from three aspects: natural aesthetic and spiritual significance, simple ecological environmental protection consciousness, and life community. They reveal the true meaning of beauty in nature, interpret the beauty of harmony in harmony with nature, advocate returning to nature and the beautiful nature of human beings, and open up a natural path leading to truth, goodness, and beauty for people to pursue their spiritual home. In addition, they also expressed their deep concern for natural resources and the natural environment and called on people to respect life and protect and rationally use natural resources. It highlights that people are not the real masters of the nature, but as an inseparable member of the nature, they form an equal community of destiny with other creatures in the world. The value of British and American romantic literature lies in revealing the deep relationship and mutual influence between human beings and nature and prompting people to comprehend the importance of protecting the ecological environment and living in harmony with nature.

## 1. Introduction

At the end of the 19th century, due to the changes in nature, human beings began to pay more and more attention to the external living environment, thus generating a new perspective to look at the relationship between human and nature and ecological consciousness [1]. “Ecological consciousness is a special value concept, which is based on the mutual relationship between all ecology and human activities in nature, including itself [2]. It reflects the new relationship between man and nature—the viewpoint and theory of harmony between man and nature and the sum of emotions [3].” Romantic literature lays a foundation for the expansion of modern ecological thought by paying attention to natural beauty, loving nature and returning to nature itself [4]. Therefore, the romantic tradition of literature has always played a genetic role in the reproduction of ecological thought. British and American romantic literature eulogizes the beauty of nature and writes that nature is an organic and unified whole, which stimulates people's ecological awareness of advocating, integrating, and respecting nature [5]. In the doubt of the rapid growth of the industrial society, under the obvious unreasonable utilization of resources and the pollution of the natural environment, the British and American romantic culture has grown rapidly and produced strong characteristics of the post industrial society [6]. It contains rich and precious environmental awareness information, and reflects the real concern of British and American romantic writers for the natural ecology. Table1 compares the characteristics of romanticism, realism, and modernism [7].

The article "The Ecological Consciousness of Natural Writing in British and American Romantic Literature" was retracted in 2023. Reasons: unreliable results or conclusions; concerns about the data; concerns about the peer review; concerns about the citations.

From the end of the 18th century to the thirties of the 19th century, romanticism was deeply disappointed by the “Kingdom of reason” designed by French Enlightenment philosophers, and tried to seek new spiritual support (1) content: no longer deliberately highlighting human philosophical rationality, but deeply exploring human emotional world (2) style: imagination-based and ups and downs of French Hugo's Notre Dame de Paris; The liberation of Prometheus by Shelley; Heine's Germany, the legend of winter [8]. Nature plays an important role in British and American literature. The development of British and American ecological culture cannot be separated from the new romantic cultural movement at the end of the 18th century and the beginning of the 19th century. It plays a very important role in British and American culture. The appearance of the beauty of art has always been the proof of people's yearning for a harmonious ecological “Utopia.” The emphasis on natural beauty in literature itself has also laid a foundation for the expansion of human ecological consciousness. In human ecological culture, natural scenery is the extension of human perceptual existence, and the externalization of human richness and human existence has formed a perfect and harmonious aesthetic order [9]. However, in the era of social development with a relatively long human history, the ecological crisis has been caused by the contradiction between man and nature and the trend of replacing the whole ecological world by human society. For a long time, few people in the literature have reflected on the consequences of human conquest of nature [10]. In the view of romantic writers, nature is the organic integration of man and nature, and nature is the soul of man. Therefore, all cultural exploration and cultural discussion cannot ignore the theme of the post industrial revolution period, which has strong characteristics of the times and the romantic tradition of the British and American ecological culture [11]. British and American ecological literature has far-reaching ideological roots. Although the Western mainstream culture as a whole believes in anthropocentrism and the idea of conquering, transforming, and utilizing nature, we can still find clues to the development of ecological thinking [12]. The romantic tradition of literature has always played an important role in the reproduction of ecological thinking. The “gene” role: The romantic view of nature is based on the industrial revolution of the 18th century and the environmental destruction it caused, and it is the abhorrence of industrial civilization. It liberates people from the shackles of various social customs and social morals, the individual is fully respected, the value identity of the group is abandoned, and the absolute truth of reason is doubted. Therefore, people always see some real images of subjective imagination, such as torrents, cliffs, storms, forests, and strange landscapes. In this respect, Wordsworth has the following expression: “I generally choose the theme of simple and idyllic life. Because in this life, the main impulses of people's hearts have been well cultivated, and they can obtain a more mature psychological state, reduce a little restraint, and speak more concise and powerful words. Finally, it is precisely because in this life, people's passion is a beautiful and eternal form of nature” [13].

The article "The Ecological Consciousness of Natural Writing in British and American Romantic Literature" was retracted in 2023. Reasons: unreliable results or conclusions; concerns about the data; concerns about the peer review; concerns about the citations.

## 2. Theoretical Research

### 2.1. Romantic Ecology

“Romantic ecology” has now become a term widely used by ecocritics. Looking back at the green research in the British and American circles, outside the academic circle of literary criticism, the earlier research on British and American romanticism under the name of “Romantic Ecology” was the work of American environmental historian Donald Worcester in “Natural Nature.” The book Economic Systems: A History of Ecological Thought (1977) [14] was so influential that it was published three times in the 1970s, 1980s, and 1990s. The “romantic ecology” used by the author in this book mainly refers to the ecological thought of American transcendentalist writer Thoreau, as well as the ecological thought of British and German romantic writers. The most direct connection between Romanticism and ecology, according to Worcester, is in the Romantic's way of looking at nature, which is “essentially ecological, that is, he considers relationships, dependencies, and holistic qualities.” In addition, both share common subversive/critical goals: “established concepts formed by science,” “values and structures of ever-expanding capitalism,” and “traditional prejudices of Western religions against nature” [15].

The article "The Ecological Consciousness of Natural Writing in British and American Romantic Literature" was retracted in 2023. Reasons: unreliable results or conclusions; concerns about the data; concerns about the peer review; concerns about the citations.

Therefore, people always see some real images of subjective imagination, such as torrents, cliffs, storms, forests, and strange landscapes. In this respect, Wordsworth has the following expression: “I generally choose the theme of simple and idyllic life. Because in this life, the main impulses of people's hearts have been well cultivated, and they can obtain a more mature psychological state, reduce a little restraint, and speak more concise and powerful words. Finally, it is precisely because in this life, people's passion is a beautiful and eternal form of nature” [16]. Bate takes Wordsworth as an example to reflect on the ecological thinking of romantic poetry, and points out that Fahrenheit does not examine nature from the traditional “enlightenment perspective,” nor does the poet regard nature as something that is tamed, controlled, and exploited, but a person. He hopes that through the understanding of nature, readers will find that life is in a system that has a subtle relationship with nature, so as to explore the position of people in this system [17]. Therefore, Bate said that Wordsworth became the first true nature poet in the United States, representing a good and continuous concept of the integration of man and nature. Wordsworth's natural concern is also an environmental concern, and his politics is also a “green politics.” In Bate's eyes, this concept of romantic poetry has had a great impact on the subsequent resource conservation movement and has a considerable impact on the current problem of dealing with environmental protection crisis [18].  Figure 1 shows the management system of environmental protection and the measure.

Bett's second work on romantic ecology, “Song of the Earth,” still interprets the text in an “ecological context,” but the text has expanded to include modern and contemporary works in Britain and America, from Jane Austen to Elizabeth, Bishop, and then to Gary [19]. In this book, Bate reemphasizes that romantic literature's love of nature, strong individualism, and political activism made it suitable for sowing the seeds of the green movement [20]. Bate also reevaluated Wordsworth's aesthetics of the sublime, arguing that the sublime was not egoistic, but ecological. Following Bethe, especially from the mid-1990s when “ecocriticism” came into being, critics in Britain and America developed the study of “romantic ecology”. Ecocritics have different emphasis on romantic ecology. These research results have a greater impact, as well as the book “Green Writing: Romanticism and Ecology” published by the British critic James McKusick in 2000. The book uses “ecology in romantic works” to summarize “a new concept of the relationship between man and the natural world” created by the British romantic poets. The most important points of this environmental theory are “species adaptation of habitats”, “interconnectedness of all life forms” and “potential catastrophic impact of human intervention on natural systems.” It is pointed out in this book that it is these reunderstandings of Chinese romantic poets that have caused a great impact on Chinese environmental writers in the 19th and early 20th centuries. It is precisely this kind of Chinese romantic environment that they are concerned about. Therefore, he put forward the “ecological process review” completely and clearly put forward the viewpoint of China's wilderness areas.  Table 2 lists the main ecological problems in my country and the main reasons for the ecological problems. McCusick took Coleridge, Wordsworth, John Clare, William Blake, Emerson, Thoreau, Muir, Mary Austin, and other British and American romantics as righteous poets and writers of nature writing. All are placed in the “green writing” category of “romantic ecology.” He also emphasized the inherited relationship between British and American Romantic thought.

The article "The Ecological Consciousness of Natural Writing in British and American Romantic Literature" was retracted in 2023. Reasons: unreliable results or conclusions; concerns about the data; concerns about the peer review; concerns about the citations.

So how to define “romantic ecology”? With reference to the abovementioned relevant writings, the author believes that “ecology” in “romantic ecology” does not refer to a scientific theory, but a literary ecological thought. It generally refers to the cultural environment knowledge contained in British and American romantic literature, but it can also be used to explain this concept reflected in other poetic texts. Specifically, the main contents of romanticism ecology are advocating the natural view of organic system and opposing the mechanical natural view. In the author's attitude of respecting nature, there is also the author's ecological ethics spirit of deeply caring for nature; however, the author's creation about nature in the novel does not take the nature as the background but emphasizes the significance of the nature itself, and uses this creation to express his criticism of the ills of modern industrial society, and also shows his positive thoughts on the construction of modern human society.

### 2.2. Ecocriticism

Environmental Criticism and environmental research are critical concepts. This view began in China in the late 1980s and Britain in the early 1990s. However, as a research field, environmental criticism first occurred in the late 1970s. Nevada Institute, Reno, should be considered as an important cradle of American cultural ecological criticism. The American Society of Western culture, founded in 1965, is also interested in studying Western culture. Michael P. Branch, now a professor of literature and the environment at the University of Nevada, Reno, in his paper “What is Ecocriticism?” presented at the society's conference in the late 1970s, put “ecocriticism.” The use of the term dates back to William Rueckert's 1978 “Literature and Ecology: An Experiment in Ecocriticism,” which refers to the early 1970s. Writing on the environmental crisis, aiming at applying ecology and ecological concepts to the study of literature, it tentatively highlights the theme of literature and ecology, and William Rueckert is considered to be the first person to use the concept of “ecocriticism.”

The article "The Ecological Consciousness of Natural Writing in British and American Romantic Literature" was retracted in 2023. Reasons: unreliable results or conclusions; concerns about the data; concerns about the peer review; concerns about the citations.

The terms “ecocriticism” and “ecology” seem to have died down in the field of literary criticism. It was not until the 1989 Western Conference on American Literature that Cheryl Grotferty, then a Ph.D. student at Cornell University, not only revived the term “ecocriticism,” but pushed the term to radiate to what had been previously a field called “Nature Writing Studies.” Grotferty later became a professor of literature and the environment at the University of Nevada, Reno, and played a pivotal role in the creation of American ecocriticism. In 1996, she and From co-edited “Ecocriticism Reader: Milestones in Literary Ecology,” and she was also one of the main founders when the Literary and Environmental Research Society was established in 1992. Another person who played an important role in the establishment of American ecocriticism was Slovic. He has been a professor of literature and a lecturer of environmental scholars at the University of Nevada, Reno University, and Idaho College. He is also the cofounder of the Chinese literature and Environmental Science Research Association. President, Slovic, has been the founding editor of the journal “Interdisciplinary Research on Literature and Environment” since its establishment in 1993. Thus, through rapid growth, by the early 1990s, China's ecological criticism had formed a brand-new professional type and an effective professional operation mechanism, including professional journals and formal professional institutions. What is interesting is that the American Ecological Criticism movement is mainly generated in the universities in western California, because these schools are often far away from the major academic authorities in the big cities of the United States and the east and west coasts, and more dependent on the good research system and academic atmosphere of the pluralistic and democratic development of the United States.

The article "The Ecological Consciousness of Natural Writing in British and American Romantic Literature" was retracted in 2023. Reasons: unreliable results or conclusions; concerns about the data; concerns about the peer review; concerns about the citations.

The ecological comments in the United States are mainly based on environmental culture. Ecological criticism is not a simple theoretical deduction, and environmental culture is also the source of ecological criticism. The ideological origin of ecological criticism can be traced back to three American novelists in the 19th century. They are Emerson, Fuller, and Thoreau. They all sing about nature, the power of life and the wilderness. They are all extraordinary writers. The innovation of Emerson's view of nature is to highlight the loftiness and profundity of nature, oppose the contradiction between man and nature, and advocate the mutually beneficial coexistence of man and nature. As a transcendentalist writer, Emerson emphasized that man communicated with nature through spirituality and believed that human beings could not fully accept the beauty of nature. This positively influenced subsequent environmental literature and ecocriticism in the United States.  Figure 2 is an analysis of the problems and measures of how to make people and nature coexist in harmony in building a beautiful China.

## 3. Analysis of Ecological Consciousness in British and American Romantic Literature

### 3.1. The Aesthetic and Spiritual Significance of Nature

“Respect for nature” is an important idea in romantic art. Some of the “reverence for nature” stems from human's natural attachment to nature, while others stem from various disadvantages and pressures brought about by the development of industrial civilization. One of the common characteristics of modern English literature and poetry is to use nature as a carrier to express emotions. Wordsworth was a pioneer of modern British romantic culture. He was tired of the noise of the city. From 1799, he retired to his hometown; namely, the nature of the mountains in the lake area has lasted for more than 50 years. Wordsworth believes “Nature has some powers that can make people's hearts infected, and nature will move people with tranquility and beauty, and can lead people to joy. For example, the most ordinary flowers can also inspire people's inspiration, and daisies can teach people to live in Rekindling hope in times of distress, daffodils can heal the wounds of people's hearts.” Obviously, Wordsworth did not simply sing the praises of nature, but inspired people's spiritual realm through the description of nature, inspired people's spiritual growth, and sought for human achievement. “The Return of Inner Nature” is the central theme of his poetry.

Wordsworth wrote a lot of romantic idyllic poems in harmony with nature in his life. Natural objects presented an independent aesthetic character in his poems and for the first time truly became the object of human aesthetics. In this way, a new kind of natural gospel and ecological awareness can be embodied. Wordsworth is like a harp that will play harmonious music when the wind blows. The grace and rhythm of all things in nature will knock on the door of his inspiration in time. Acura has naturally become the most important mission of his poetry creation. The world written by the author is naturally a social world integrating human nature and divinity. Wordsworth's ultimate goal is to explore the psychological impact of nature on people through his detailed description of natural scenery. Human life is undergoing great changes in a social order gradually destroyed by traditional rationality, survival methods, and values. Life contains risk, stress, and anxiety. People's original good nature began to weaken slowly. The direct result is that our cultural life is becoming more and more vulgar and impetuous, and materialism and utilitarianism are prevailing. Wordsworth lives in this noisy city. He can only get inner peace by hiding from nature.

The article "The Ecological Consciousness of Natural Writing in British and American Romantic Literature" was retracted in 2023. Reasons: unreliable results or conclusions; concerns about the data; concerns about the peer review; concerns about the citations.

Nature “gave him a warm feeling, restored my peace, let me forget the unhappiness of life, and a kind of peace and warmth led me forward.” The author is very happy because “I found the nanny of my soul in nature, guiding and protecting the soul of my whole moral life.” Industrial civilization has become a way of suppressing and stifling human nature, and people have gradually lost their ability to appreciate the “sunrise and sunset” state of mind. This is a basic spiritual misfortune. Nature is the embodiment of human truth, goodness, and beauty. It can not only purify people's soul but also cultivate people's moral character. Only by respecting nature and returning to nature can people return to the beautiful nature on earth.  Figure 3 shows the public participation in the protection of the natural environment in my country. Tinden Abbey can be said to be a new romantic hymn, which embodies Wordsworth's profound meaning of respecting nature, actively integrating into nature, and deeply feeling the great impact of nature on human spirit. In lyrical ballads, Wordsworth wrote a lot of ecological poems to praise the harmonious interpersonal relationship between heaven and man. It requires people to “repair people's discrimination ability, and realize beautiful integration with the universe under the condition of loving and being close to nature.” Wordsworth's romantic poetic view of nature expresses his profound philosophical thinking on the relationship between heaven and man, and has profound practical significance.

The article "The Ecological Consciousness of Natural Writing in British and American Romantic Literature" was retracted in 2023. Reasons: unreliable results or conclusions; concerns about the data; concerns about the peer review; concerns about the citations.

### 3.2. Simple Ecological Awareness

Cooper is known as the pioneer of American literature and the first American writer to achieve worldwide fame. Cooper had an innate affinity for nature from childhood, fascinated by the lakes, forests and legends of the Indians near his home. He roamed the banks of rivers, wandered in forests, observed all kinds of people and things in the world with cold eyes, and thought about the true meaning of life. Bo is the central character and reflects the life of the western frontier of the United States in the “Leather Socks” five parts, namely, “The Pioneers,” “The Last of the Mohicans,” “The Prairie,” “The Pathfinder,” and “The Deer Killer.” Romance stories are popular. “Leather Socks” Nati Bangpo lives in the virgin forest, abides by forest laws, is familiar with hunting skills, respects nature, respects all life in nature; as a hunter, he said frankly: “In my opinion, if the first deer, it's a sin to shoot the second deer before it's finished eating.” He had a dignified demeanor and was devoted to nature. When he saw Lin Ru and God, he fled all the way to the west, trying to stay away from the axe of civilized villages and towns. Cooper hopes that his works can represent “the reality of early human civilization.” He reflects the mysterious native forests, rivers, creeks, cliffs, mountains, cliffs, and huge waterfalls in western California, and connects the appearance of the wild world with the life of primitive forest residents in the nature. The story unfolds according to this description: ”in a huge mountain near the center of New York State, the undulating peaks and occasional stones add color to the original romantic and picturesque scenery. The river flows through the long, fertile mountain streams. Everywhere is full of vitality.” In addition, it also shows the man-made landscapes that prove the historical value of the American frontier, such as the British colonial fortress and the dome cement houses carefully built by the Indians. These mud houses are flanked by lakes or built in water. The work contains a simple and strong North American flavor, showing a picture of natural ecological harmony that has not been invaded by industrial civilization, and is full of the beauty of natural harmony of the original ecology.  Table 3 shows the ecological protection measures adopted by my country for different ecological systems.

## 4. “Community of Life” in British and American Romantic Ecology Literature

Emerson's transcendental view of nature has influenced many American writers. Thoreau, the pioneer, is one of the greatest ecological novelists in the post romantic literature period. Walden lake is a classic work written by Thoreau, a scientific pioneer, based on his living experience in the primeval forests of the United States. The main idea of Walden lake is to explore knowledge about the relationship between his life and nature. In this book, the description of nature is also very rich. It is the pinnacle of Thoreau's ecological thinking and an important milestone in the history of American literature. His exquisite and unique natural ecological theory has greatly inspired future generations. British nature critic Boyle once pointed out: “Thoreau showed us a kind of non-human existence, a survival beyond other members of the world, and showed the significance of all existence in the great nature, including the human body.” Thoreau was alone in living in the virgin forest on the banks of Walden Pond, surrounded by towering ancient trees, green lake water, birds, and beasts, is a primitive scene. It is no wonder that Emerson compared Thoreau to the simple and straightforward Adam, which is very vivid. In “Walden,” Thoreau expounded two aspects of content, one is all things in nature, and the other is that modern people should return to simplicity and nature. Thoreau once said in Walden Lake: “I went to the jungle because I wanted to live in a free and simple way. Only facing the most real things in life, it depends on how I can understand what life means to me. Only in this way, when I die, I will not find that I have not really lived. I want to live deeply and absorb the vitality of life.” Figure 4 shows the 2010–2020 scholars studying Thoreau and the trend of man and nature development.

The article "The Ecological Consciousness of Natural Writing in British and American Romantic Literature" was retracted in 2023. Reasons: unreliable results or conclusions; concerns about the data; concerns about the peer review; concerns about the citations.

From ancient times to the present, human beings have always been looking for the meaning of life and life. Thoreau took a road of returning to the pure life of human primitive times. Although that kind of life may seem rough or even very simple, it is precisely the way that is closest to nature and the best way to make people feel the existence of life. Human life is connected with nature, but it is always an important part of nature. Human life always shares the beauty of nature with the sun, moon, and stars. All human activities that deviate from nature are violations of human nature. Like other thinkers, Thoreau was also closer to nature and liked nature more, and he was more sensitive to the power and influence of nature. This experience had an important impact on the maturity of Thoreau's thinking. In the process of implementing Emerson's Transcendentalism, Thoreau further developed the transcendental natural science concept into a real biological and ecological consciousness. As a person who loves and values nature, he further clarified that man is not the real master of nature. Compared with anything, human beings are inseparable members in nature, and together form an equal survival community of the universal blood family, as shown in Figure 5. The connection between man and nature in a broad sense. Thoreau believes that the modern people's wanton plundering of resources has made people gradually lose their material homes, and the unbalanced development of society has caused people's spiritual plight. The core of the romantic view of nature is a view that later people regarded as ecology—the exploration of the concept of the integrity or interconnectedness of life in the universe, emphasizing the interdependence and interconnection between humans and natural objects. The romantic desire for this holistic thought is indescribable.

The article "The Ecological Consciousness of Natural Writing in British and American Romantic Literature" was retracted in 2023. Reasons: unreliable results or conclusions; concerns about the data; concerns about the peer review; concerns about the citations.

## 5. Conclusion

Writers in the era of British and American romantic literature are keen to eulogize nature, and there is a good cultural tradition in their literature, which is the integration of the ecological concept of “loving and respecting nature.” Therefore, they are also widely regarded by Western critics as literary groups with strong ecological consciousness, and the relationship between nature and human beings is also the main theme discussed in their literature. For children, the writing of nature is not a simple expression of the external scenery, and the interaction between children and nature is also colorful, showing children's concern for emotion, consciousness, humanities, and other fields. Because nature does not belong to man, and man also belongs to nature. The discussion of the relationship between man and nature is always a manifestation of mankind's pursuit of a harmonious ecological life. It aims to awaken people to restore the natural characteristics of human life and guide people to truly appreciate nature. The eternal beauty contained in it is value and truth. The significance of romantic poetry is undoubtedly to discover the profound connections and interactions between human social relations, integrate them into human spiritual and conscious activities, strive to restore the harmonious feelings of human beings towards nature, and integrate these feelings into all aspects of people's daily life and culture, thus helping human beings rerealize the necessity of harmonious coexistence with the natural environment and nature. Meaning is in this sense, romantic poetry has finally moved towards eternity.

## Figures and Tables

**Figure 1:** Environmental protection system and measures.

**Figure 2:** Problems and measures for the harmonious coexistence of man and nature.

**Figure 3:** Investigation and analysis of the types of organizations participating in public environmental protection activities.

The article "The Ecological Consciousness of Natural Writing in British and American Romantic Literature" was retracted in 2023. Reasons: unreliable results or conclusions; concerns about the data; concerns about the peer review; concerns about the citations.

**Figure 4:** The research trend of Thoreau's “man and nature.”

**Figure 5:** The connection between man and nature in a broad sense.

**Table 1:** Comparison of the characteristics of romanticism, realism, and modernism.

	Background	Features	Represent
Romanticism	From the end of the 18th century to the 1830s, people were deeply disappointed with the “realm of reason” envisioned by enlightenment thinkers and struggled to find new spiritual sustenance	(1) Content: no longer deliberately highlights the rationality of human beings, but deeply explores the emotional world of human beings (2) Style: mainly imaginative ideas and ups and downs	“Notre Dame de Paris” by Hugo, France: “Prometheus Liberated” by Shelley, England: “Germany, a Winter's Fairy Tale” by Heine Deutsche

Reality Lord	After the 1830s, the social contradictions in European and American capitalist countries became increasingly acute	Pays attention to social issues, typically reproduces social features, deeply analyzes the nature of social life, and exposes and criticizes social evils	French Balzac's “Human Comedy”; Russia's Leo Tolstoy's “Anna Karenina”, etc.

Modernism	The two world wars, the capitalist world economic crisis in the 1930s, and serious social problems showed the social spiritual crisis	Concentrated self-expression: bizarre creative techniques: Blurred story background, unclear causal relationship, language style deviating from biography	The Old Man and the Sea by Hemingway and Waiting for Godot by Beckett

**Table 2:** My country's main ecological problems and their causes.

Area name	Major ecological issues	Cause of formation	
A	Deforestation, soil erosion, severe grassland degradation	Natural background	Man-made causes
B	Severely degraded grassland	Semiarid steppe area	Overcultivation, overcutting, overgrazing are serious
C	Severe soil erosion	Less precipitation, drier climate	Serious overgrazing
DE		Warm temperate subhumid areas	Densely populated
F	Major ecological issues	Subtropical hills, abundant rainfall	People live in poverty, overcultivation, overcutting
G		Subtropical hilly and mountainous areas with complex geological conditions	Ecologically fragile due to climate change and human activities

**Table 3:** Conservation measures for different ecosystems.

Ecological zoning	Environmental element status			Utilization and protection measures
Crisis zone	Atmosphere	Waters	Soil vegetation	Development should be completely limited and no human pressure should occur, and comprehensive nature conservation measures should be implemented
	x	x	x	
	±	x	x	
	x	±	x	

Unfavorable zone	x	x	±	Development should be limited, and human pressure should be reduced for unfavorable environments, and targeted natural protection measures should be implemented
	x	±	±	
	±		±	
	±	±		
	−	−	−	

Stable zone	−	−	+	To stabilize artificial pressure on environmental claims and implement natural conservation measures applicable to them
	−	+	−	
	+	+	+	
	−	+	+	

Favorable area	+	−	+	Limits of anthropogenic pressure need to be specified, and natural conservation measures determined as needed
	+	+	−	

The article "The Ecological Consciousness of Natural Writing in British and American Romantic Literature" was retracted in 2023. Reasons: unreliable results or conclusions; concerns about the data; concerns about the peer review; concerns about the citations.

## Data Availability

The labeled data set used to support the findings of this study is available from the corresponding author upon request.

## References

[1] Guslyakova A. V., Guslyakova N. I., Valeeva N. G. (2020). Ecological consciousness of the XXI century human and the ways of its verbalization in the media discourse environment. *Rudn Journal of Ecology and Life Safety*.

[2] Gangwar D. S. (2020). Cultivation of ecological consciousness for a sustainable agroecosystem. *Journal of International Business Studies*.

[3] Toktosunova A. I., Alym Baeva T. B. (2021). Chinghiz Aitmatov about a precipice between people and alive suffering nature and the formation of ecological consciousness. *Historical and Social-educational Ideas*.

[4] Wang Y. (2020). Hemingway’s ecological consciousness in “an African story”. *Journal of Language Teaching and Research*.

[5] Sorokoumova E. A., Cherdymova E. I. (2021). Developing structural components of ecological consciousness to promote civic identity formation. *Psychological Science and Education*.

[6] Barman D. M. (2020). Ecological consciousness and self-realization-- an identification: a step towards spiritualistic world. *Global Journal of Science Frontier Research*.

[7] Krasilnikova E. V., Kuznecova S. N. (2021). On the formation of environmental consciousness among students of an agricultural university. *IOP Conference Series: Earth and Environmental Science*.

[8] Bhandari R. (2022). Deep ecological consciousness and interconnectedness in William wordsworth€s Tintern Abbey. *Technium Social Sciences Journal*.

[9] Sullivan G. (2017). *Runaway: Gregory Bateson, the Double Consciousness Bind, and the Rise of Ecological*.

[10] Raftopoulos M. (2020). Rural community-based tourism and its impact on ecological consciousness, environmental stewardship and social structures. *Bulletin of Latin American Research*.

[11] Andráscsai O. (2021). Ecological consciousness and value orientations in business. *Ecologically Conscious Organizations*.

[12] Sarah R. (2022). Raven’s land: American literary history in medias res. *American Literary History*.

[13] Song C., Buysse A., Zhang W. (2020). Coping with minority stress in romantic relationships among lesbian, gay and bisexual people. *Current Psychology*.

The article "The Ecological Consciousness of Natural Writing in British and American Romantic Literature" was retracted in 2023. Reasons: unreliable results or conclusions; concerns about the data; concerns about the peer review; concerns about the citations.

[14] Qi L. (2021). Women’s voices in the victorian era – feminist consciousness in the bronte sisters’ works. *Journal of Contemporary Educational Research*.

[15] Munroe J. (2021). The marvels of the world: an anthology of nature writing before 1700. *Interdisciplinary Studies in Literature and Environment*.

[16] Zhang H., Qi C. (2021). Impact of environmental and health consciousness on ecological consumption intention: the moderating effects of haze and self-competence. *Journal of Consumer Affairs*.

[17] Kaushik R. (2021). Literature, ontology, and implex in merleau-ponty: writing and finding the concrete limit of phenomena humanities. *Humanities*.

[18] Burke M., Coates K., Wales K. (2022). Charles dickens, children’s author: narrative as rhetoric in a child’s history of England. *Language and Literature*.

[19] Christine B., Lucas A., Dietrich (2022). *Writing Across the Color Line: U.S. Print Culture and the Rise of Ethnic Literature, 1877–1920*.

[20] Xiao-Qin X. U. (2020). Cultivation of reading, writing, and critical thinking in the teaching of selected readings in American literature. *Chinese and American English Teaching: The English Version*.

